# Artificial Liver Support System Combined with Liver Transplantation in the Treatment of Patients with Acute-on-Chronic Liver Failure

**DOI:** 10.1371/journal.pone.0058738

**Published:** 2013-03-14

**Authors:** Xiao Xu, Xiaoli Liu, Qi Ling, Qiang Wei, Zhikun Liu, Xiaowei Xu, Lin Zhou, Min Zhang, Jian Wu, Jianrong Huang, Jifang Sheng, Shusen Zheng, Lanjuan Li

**Affiliations:** 1 Key Lab of Combined Multi-Organ Transplantation, Ministry of Public Health, Division of Hepatobiliary and Pancreatic Surgery, Department of Surgery, First Affiliated Hospital, Zhejiang University School of Medicine, Hangzhou, Zhejiang, China; 2 State Key Laboratory for Diagnosis and Treatment of Infectious Diseases, First Affiliated Hospital, Zhejiang University School of Medicine, Hangzhou, China; The University of Hong Kong, Hong Kong

## Abstract

**Background:**

The search for a strategy to provide temporary liver support and salvage the patients with acute-on-chronic liver failure (ACLF) remains an important issue. This study was designed to evaluate the experience in artificial liver support system (ALSS) combined with liver transplantation (LT) in the treatment of ACLF.

**Methodology/Principal Findings:**

One hundred and seventy one patients with HBV related ACLF undergoing LT between January 2001 and December 2009 were included. Of the 171 patients, 115 received 247 sessions of plasma exchange-centered ALSS treatment prior to LT (ALSS-LT group) and the other 56 received emergency LT (LT group). The MELD score were 31±6 and 30±7 in ALSS-LT group and LT group. ALSS treatment resulted in improvement of liver function and better tolerance to LT. The average level of serum total bilirubin before LT was lower than that before the first time of ALSS treatment. The median waiting time for a donor liver was 12 days (2–226 days) from the first run of ALSS treatment to LT. Compared to LT group, the beneficial influences of ALSS on intraoperative blood loss and endotracheal intubation time were also observed in ALSS-LT group. The 1-year and 5-year survival rates in the ALSS-LT group and LT group were 79.2% and 83%, 69.7% and 78.6%.

**Conclusions/Significance:**

Plasma exchange-centered ALSS is beneficial in salvaging patients with ACLF when a donor liver is not available. The consequential LT is the fundamental treatment modality to rescue these patients and lead to a similar survival rate as those patients receiving emergency transplantation.

## Introduction

Liver failure remains a disease associated with high mortality. In China, because of the high prevalence of hepatitis B, hepatitis B virus-related acute-on-chronic liver failure (ACLF) is a common cause of liver failure, which is much different from the western countries where drugs, alcohol, and hepatitis C are the major causes. According to Asian Pacific Association for the Study of the Liver, ACLF has been recently defined as ‘acute hepatic insult manifesting as jaundice and coagulopathy, complicated within 4 weeks by ascites and/or encephalopathy in a patient with previously diagnosed or undiagnosed chronic liver disease [1].

Liver transplantation (LT) is the best treatment for salvaging patients with ACLF. However, LT is not always possible because of donor shortage. Enormous attempts at providing temporary liver support have been made, with an aim to increase survival rate or improve the condition of the patient until a donor is available. In the past decades, a variety of artificial liver support system (ALSS), including plasma exchange (PE), hemoperfusion, PE plus continuous hemodiafiltration, MARS and fractionated plasma separation, adsorption and dialysis system, have been employed in the management of liver failure [2].

Our previous study has demonstrated that ALSS can efficiently decrease the mortality of patients with severe hepatitis of early and middle stages [3]. However, for patients with ACLF, since hepatocytes undergo massive denaturation, necrosis and dysfunction, it is difficult to completely reverse the clinical course of the disease with routine medical management and even combined with ALSS. Under this circumstance, LT is usually indispensable. In the present study, we described our experience of PE-centered ALSS combined with LT in the rescue of patients with ACLF.

## Methods

### 2.1 Patients

This study was approved by the First Affiliated Hospital, Zhejiang University School of Medicine and the current regulation of the Chinese Government, and the Declaration of Helsinki were strictly followed for each organ donation and transplant performed in our center. Written informed consents from each donor and recipient were obtained. No donor livers were harvested from executed prisoners. All the data was analyzed anonymously.

From January 2001 to December 2009, 796 patients underwent LT at our hospital. United Network for Organ Sharing status was used as the organ allocation system before December 2002, and Model for End-Stage Liver Disease (MELD) score was applied after January 2003. Their primary diseases included hepatic malignancies (n = 310) and benign end-stage liver diseases (n = 486). Malignancies, retransplantation, and combined transplantation were excluded. Among the 486 cases of benign end-stage liver diseases, 171 cases of ACLF with a known history of chronic hepatitis B or cirrhosis were finally enrolled in this retrospective study. Of these 171 cases, 115 received 247 sessions of ALSS treatment before LT (ALSS-LT group), whereas the other 56 cases fortunately gained appropriate donor livers and received emergency LT within 72 h after their referral to our centre, without any prior ALSS treatment (LT group). The baseline characteristics including age, gender, serum total bilirubin, MELD scores, and major complications of the above two groups were collected at the time of admission and summarized in Table 1. MELD score was calculated as 9.57×log_e_ (Cr mg/dl)+3.78×log_e_ (TB mg/dl)+11.20×log_e_ (international normalized ratio)+6.43 [4]. Lamivudine combined with low-dose intramuscular hepatitis B immunoglobulin therapy was applied in all patients [5]. Immunosuppressive regimen was triple therapy incorporating tacrolimus or cyclosporin A, mycophenolate and steroid [6].

**Table 1:** The baseline patient characteristics.

	ALSS-LT group (n = 115)	LT group (n = 56)	*P* value
Age (years)	46±10	45±10	NS
Gender (male/female)	100/15	45/11	NS
TB ( µmol/L)	557±195	537±201	NS
MELD score	31±6	30±7	NS
Infections	33	15	NS
Encephalopathy	54	24	NS
Hepatorenal syndrome	29	12	NS

Abbreviations: ALSS, artificial liver support system; LT, liver transplantation; TB, total bilirubin; MELD, model for End-Stage Liver Disease; HBV, hepatitis B virus.

### 2.2 ALSS treatment

Blood access was established through a double-lumen catheter via the patient's jugular or femoral vein. The methods of ALSS included PE, plasma perfusion, continuous hemodiafiltration and MARS. PE was performed with plasma separator Plasmacure PS-06 (Kuraray Co., Tokyo, Japan). The total volume of exchanged plasma was about 3300 ml, and the exchange rate of plasma was 22–25 ml/min. Continuous hemodiafiltration was performed with Diafilter D-30NR (Minntech Co., Minneapolis, MN). Plasma perfusion utilizing Adsorba 300C contained 300 g cellulose coated charcoal (Gambro Dialysatoren GmbH Co., KG, Hechingen, Germany). The MARS system (MARS monitor, Teraklin AG, Rostock, Germany) was used, and its albumin circuit, containing 600 mL 20% human albumin, was driven at 150 mL/min. Dexamethasone (5 mg) and prophylactic antibiotics were routinely given. Totally 20–60 mg heparin and 10–30 mg protamine sulphate were given in one run of ALSS treatment.

The detailed methods of PE-centered ALSS were performed based on individuals' conditions. For example, patients with coagulopathy were indicated for PE; when the patient had hepatic encephalopathy, we used PE plus plasma perfusion or continuous hemodiafiltration. For patients complicated with hepatorenal syndrome or imbalance of water or electrolytes, we applied PE plus continuous hemodiafiltration or MARS. In ALSS-LT group, 247 sessions of ALSS were applied to 115 patients, with PE 162 times, PE plus plasma perfusion 52 times, PE plus continuous hemodiafiltration 18 times and MARS 15 times.

### 2.3 Data Collection

Patient demographic, surgical, and postoperative data were collected by chart review and from surgical records. Serum parameters of serum total bilirubin, alanine aminotransferase, aspartate aminotransferase, total bile acid, creatinine, prothrombin time and electrolytes were closely monitored before and after every session of ALSS treatment or during the perioperative period.

### 2.4 Statistical analysis

The values were expressed as mean±SD. The data were statistically analyzed by SPSS 10.0 software package (SPSS Inc, Chicago, IL). The laboratory data were compared by Wilcoxon's rank-sum test or Mann-Whitney U test. Chi-square test was used to compare categorical variables. Survival analysis was estimated using Kaplan-Meier method. A *P* value less than 0.05 was considered statistically significant.

## Results

### 3.1 Efficacy of ALSS

Before ALSS treatment, 115 patients in ALSS-LT group were in poor general condition, complicated by cachexia, fatigue, loss of appetite, abdominal distention, jaundice, hepatorenal syndrome or hepatic encephalopathy. After ALSS treatment, general conditions and clinical symptoms including spirit, sleeping, appetite, and hepatic encephalopathy were improved. The changes of main laboratory parameters in 4 subgroups of ALSS are listed in Table 2. The levels of serum total bilirubin declined markedly by almost 50% on average in all subgroups. PE plus continuous hemodiafiltration and MARS obviously decreased serum creatinine level with the removal rates of 45±9% and 28±4%, respectively. Prothrombin time decreased significantly in PE involved ALSS subgroups (*P*<0.05).

**Table 2:** Changes of key laboratory parameters pre- and post-artificial liver support system (ALSS) treatment in different subgroups.

Parameters	PE (n = 162)	PE+continuous hemodiafiltration (n = 52)	PE+Plasma perfusion (n = 18)	MARS (n = 15)
TB				
Pre-treatment ( µmol/L)	575±174	530±165	558±183	511±137
Post-treatment ( µmol/L)	260±96	253±82	261±95	331±115
Removal rate (%)	55±6	52±5	54±5	34±4
*P* value	<0.05	<0.05	<0.05	<0.05
Cr				
Pre-treatment ( µmol/L)	80±19	301±102	78±15	198±43
Post-treatment ( µmol/L)	76±15	169±52	74±13	145±29
Removal rate (%)	4±5	45±9	4±4	28±4
*P* value	>0.05	<0.05	>0.05	<0.05
PT				
Pre-treatment (s)	32.4±10.3	31.6±8.0	31.2±7.7	28.4±8.4
Post-treatment (s)	20.7±3.6	22.5±6.3	23.6±5.6	30.1±8.8
*P* value	<0.05	<0.05	<0.05	>0.05

Removal rate was calculated as: (pre-treatment concentration—post-treatment concentration)/pre-treatment concentration.

Abbreviations: PE, plasma exchange; TB, total bilirubin; Cr, creatinine; PT, prothrombin time.

### 3.2 Impact of ALSS on patients' transplantability

One hundred and twenty five patients of ALSS-LT group were successfully bridged to LT after attaining proper donor organs. The average level of TB before LT was significantly lower than that before the first session of ALSS treatment (476±169 µmol/L vs. 557±195 µmol/L, *P* ***<***0.05). The average levels of MELD pre-ALSS and pre-LT were 31±6 and 29±9, but no significant difference was found between them (Table 3). The median waiting time for a donor liver was 12 days (range from 2 days to 226 days) from the first run of ALSS treatment to LT.

**Table 3:** Liver function and model for End-Stage Liver Disease (MELD) score before artificial liver support system (ALSS) and before liver transplantation (LT).

	TB ( µmol/L)	ALT (U/L)	AST(U/L)	TBA µmol/L)	MELD score
Pre-first ALSS	557±195	127±113	182±152	246±98	31±6
Pre-LT	476±169	105±80	165±207	144±108	29±9
*P* value	<0.05	>0.05	>0.05	<0.05	>0.05

Abbreviations: TB, total bilirubin; ALT, alanine aminotransferase; AST, aspartate aminotransferase; TBA, total bile acid;

### 3.3 Impact of ALSS on intraoperative blood loss and ICU staying

Compared to those in LT group, there was less blood loss during the operations and shorter endotracheal intubation time for the patients in ALSS-LT group (3941.8±1997.4 ml vs. 5058.3±2193.6 ml, ***P***<0.05; 3.3±2.6 days vs. 4.5±3.6 days, ***P***<0.05). A similar trend was observed in the average ICU staying time but the reduction was not statistically significant (9.8±4.5 days vs. 10.5±4.7 days, ***P***>0.05). (Table 4).

**Table 4:** Intraoperative blood loss, intubation and ICU staying time in the artificial liver support system (ALSS)-liver transplantation (LT) group and LT group.

	Blood loss (ml)	Intubation time (days)	ICU staying time (days)
ALSS-LT group	3941.8±1997.4	3.3±2.6	9.8±4.5
LT group	5058.3±2193.6	4.5±3.6	10.5±4.7
*P* value	<0.05	<0.05	>0.05

### 3.4 Impact of ALSS combined with LT on patients' survival

In ALSS-LT group, the survival rates of 1-year and 5-year were 79.2% and 69.7%, respectively. Compared with that in ALSS-LT group, the survival of LT group did not show significant difference, with the 1-year and 5-year survival rate of 83% and 78.6%, respectively. No significant differences in survival were found between two groups (Figure 1). However, in another cohort of ACLF patients (n = 158) receiving only conventional medical therapy (no ALSS and no LT), the 1- and 3-month mortality was 79.7% and 90.5%, respectively.

**Figure 1:** Comparison of patient cumulative survival between ALSS-LT group and LT group. (*P* = 0.406) (ALSS, artificial liver support system; LT, liver transplantation).

## Discussion

The past two decades witnessed the progress of LT [7], [8]. As the only efficient procedure to treat ACLF, LT has been applied with a perioperative mortality rate of less 3% and 1-year survival rate of exceeding 80% for recipients in some major transplant centers in China [9]. At our center, ACLF related to HBV infection has been one of the main indications of LT. The shortage of donor livers, however, will undoubtedly make the patients with critical condition lose the opportunity for LT. For those who undergo LT in a deteriorating status with cachexia and disturbance of internal environment, the outcome would be unsatisfactory. The increasing discrepancy between the number of potential candidates for LT and the number of donor livers available suggests that some therapeutic alternatives for temporary liver support to patients with ACLF should be necessary [10], [11].

Recent studies have shown that extracorporeal liver support systems could temporarily support patients' liver function, improve their preoperative condition, and enhance their tolerance to surgery, thus extending the waiting time for a donor liver as a bridge to LT [12]–[16].

As a promising liver assist system, ALSS can perform partial functions of liver, with important therapeutic potentials in various patients with hepatitis, liver cirrhosis, and acute liver failure [17], [18]. ALSS treatment seemed to reduce the mortality in patients with ACLF [19]. As an important part of ALSS, PE has been long applied in fulminant hepatic failure with aim of removing overabundant toxic substances and correcting the severe coagulopathy [20]. For removal of the hepatic encephalopathic substances such as aromatic amino acids, ammonia and middle molecules, plasma perfusion or continuous hemodiafiltration are often used with PE simultaneously [21], [22]. MARS is actually combining hemodialysis/filtration and plasma perfusion, and serves to remove albumin-bound toxins and water-soluble toxins [23]. To patients complicated with hepatorenal syndrome, PE plus continuous hemodiafiltration and MARS also helped to improve renal function. In this study, PE-centered ALSS including PE alone, PE plus continuous hemodiafiltration, PE plus plasma perfusion and MARS were applied based on individuals' conditions.

Our early study has found that non-biological artificial liver techniques can efficiently decrease the mortality of patients with severe hepatitis of early and middle stages [3]. Our results supported the favorable effects of PE-centered ALSS. Before ALSS treatment, all the patients developed pre-terminal or terminal clinical manifestations, such as hepatic encephalopathy, hepatorenal syndrome, disturbance of water and electrolytes, and other severe complications. The initial serum bilirubin level of 115 patients with ACLF in the ALSS-LT group was as high as 557±195 µmol/L and still in an increasing tendency. After treatment of ALSS, liver and renal function and coagulopathy improved evidently. Neurological improvements were found in patients with encephalopathy following repeated sessions of ALSS treatment. Disorders of the internal environment prior to LT were also corrected to a certain extent, thus facilitating improvement of patients' general condition. The result of this study suggests that for patients with ACLF who are in the waiting list for LT, ALSS should be considered as an important part of preoperative management. When a donor liver is not available, salvaging ALSS should be carried out timely to support liver function and win precious waiting time till a donor liver is available. In the present study, patients after each ALSS treatment showed marked improvement in liver function and stabilized general condition, sustaining patients' lives with a median time of nearly 2 weeks and the longest time of 226 days.

The beneficial influences of ALSS on intraoperative blood loss and ICU staying were also observed. Furthermore, it was demonstrated from our results that the combined treatment of ALSS and LT achieved the same 1-year survival rate as emergency LT which was applied to those critical patients in 72 hours. Although a prospective, randomized, and controlled trial is needed to confirm the beneficial effects of ALSS, our study has undoubtedly demonstrated the efficacy and safety of ALSS in supporting liver function and extending the waiting time for donor livers. In this regard, ALSS for ACLF patients will broaden the indications of LT, and more patients in the waiting list of LT will achieve a new life.

For ACLF patients, however, what ALSS may provide is still a transient liver function support [3], [24]. The biochemical manifestation of liver failure may relapse and approach or even exceed the level before the previous ALSS treatment [25], [26]. Therefore, for the patients who developed massive necrosis of hepatocytes and lost ability of liver regeneration, several times of ALSS and sequential timely LT were needed. Although further prospective and randomized studies should be performed, we believe that ALSS is beneficial in salvaging patients with ACLF when a donor liver is not available and LT is the fundamental treatment modality to rescue these patients.
